# Deregulated AJAP1/*β*-catenin/ZEB1 signaling promotes hepatocellular carcinoma carcinogenesis and metastasis

**DOI:** 10.1038/cddis.2017.126

**Published:** 2017-04-06

**Authors:** Jihua Han, Changming Xie, Tiemin Pei, Jiabei Wang, Yaliang Lan, Kaihua Huang, Yifeng Cui, Fengyue Wang, Jiewu Zhang, Shangha Pan, Yingjian Liang, Tongsen Zhen, Ruipeng Song, Boshi Sun, Yuejin Li, Huawen Shi, Guangchao Yang, Xirui Liu, Mingxi Zhu, Yan Wang, Keyu Li, Yao Liu, Fanzheng Meng, Fei Liao, Xianzhi Meng, Xuehui Hong, Lianxin Liu

**Affiliations:** 1 Key Laboratory of Hepatosplenic Surgery, Ministry of Education, Department of General Surgery, the First Affiliated Hospital of Harbin Medical University, Harbin, China; 2 Department of Head and Neck Surgery, The Third Affiliated Hospital of Harbin Medical University, Harbin, China; 3 Department of Gastrointestinal Surgery, Zhongshan Hospital of Xiamen University, Xiamen, China; 4 Institute of Gastrointestinal Oncology, Medical College of Xiamen University, Xiamen, China

## Abstract

Adherens junctions-associated protein 1 (AJAP1) is an integral membrane protein that is thought to function as a tumor suppressor in various malignancies. Downregulation of AJAP1 mRNA levels may predict recurrence in hepatocellular carcinoma (HCC) patients, but the underlying molecular mechanism is unknown. This was addressed in the present study by examining the role of AJAP1 in HCC cell proliferation, migration, and invasion *in vitro* as well as in human specimens and mouse xenograft model. We found that AJAP1 expression was reduced in HCC cells and human HCC tissue, which was associated with metastasis. AJAP1 overexpression inhibited HCC progression and metastasis, while its silencing had the opposite effect both *in vitro* and *in vivo*. Furthermore, AJAP1 blocked epithelial–to–mesenchymal transition by interacting with *β*-catenin and inhibiting its nuclear translocation, which suppressed zinc finger E-box binding homeobox 1 (ZEB1) transcription. These results indicate that AJAP1 inhibits HCC metastasis, and is thus a potential therapeutic target for HCC treatment.

Hepatocellular carcinoma (HCC) accounts for 85–90% of cases of primary liver cancer, which is the fifth most common malignancy and the third leading cause of cancer mortality.^1^ It is estimated that there were more than 700 000 new cases of liver cancer and deaths worldwide in 2012, with about 50% of these occurring in China.^2^ Hepatitis B and C virus infection are the main causes of HCC.^3^ Other risk factors include ingestion of aflatoxin-contaminated food, cirrhosis related to heavy alcohol consumption, and nonalcoholic fatty liver disease.^4^ Surgical resection is the most common treatment for HCC; nonetheless, the frequency of tumor recurrence and distant metastasis remains high. Clarifying the molecular mechanisms underlying HCC invasiveness and metastasis can reveal novel therapeutic targets for treatment.

Adherens junctions-associated protein 1 (AJAP1, previously known as SHREW1) is a putative tumor suppressor gene located in the 1p36 region of chromosome 1, which is a hotspot for deletions in cancer.^5^ AJAP1 expression is downregulated in several malignancies, including oligodendrogliomas,^6^ neuroblastomas,^7^ glioma^8, 9, 10^ and gastric cancer.^11^ AJAP1 is membrane protein that is thought to interact with the E-cadherin/*β*-catenin complex^12^ and CD147^13^ to inhibit cell adhesion and migration. It was recently reported that the *AJAP1* promoter is highly methylated in HCC cell lines and tissues, suggesting that decreased levels of *AJAP1* mRNA are linked to HCC recurrence.^14^

Despite the above observations, the precise role of AJAP1 in HCC progression remains unknown. This was addressed in the present study using HCC patient tissue specimens, HCC cells, and mouse xenograft model. We found that AJAP1 has a tumor-suppressor role in HCC and inhibits HCC cell proliferation and metastasis via *β*-catenin/zinc finger E-box binding homeobox 1 (ZEB1) signaling.

## Results

### AJAP1 is downregulated in human HCC, which is negatively correlated with HCC metastasis

To investigate the correlation between AJAP1 expression and HCC development, we examined AJAP1 protein expression by immunohistochemistry and western blotting. Immunoreactivity was analyzed with a tissue microarray that included 95 HCC and 20 matched normal liver tissue samples (Figure 1a). AJAP1 was highly expressed in 19 out of 20 normal liver tissue samples; in addition, AJAP1 levels were higher in early- as compared to advanced-stage liver cancer (Figure 1b). AJAP1 expression was negatively correlated with tumor size (*P*<0.05), advanced disease stage (*P*<0.01), lymph node status (*P*<0.01), and metastasis (*P*<0.05). A western blot analysis confirmed the downregulation of AJAP1 expression in HCC tissues from a different cohort at our hospital (Figure 1c). Furthermore, AJAP1 levels were lower in highly metastatic HCC cell lines, including SK-Hep-1, HCCLM3, and MHCC97H cells than in those with low metastatic potential such as SMMC7721, MHCC97L and Huh7 cells, and was highest in the normal hepatic cell line (L02), as determined by western blotting and real-time PCR (Figure 1d). These results indicate that AJAP1 expression is negatively correlated with HCC metastasis and poor prognosis in patients.

### AJAP1 suppresses HCC cell proliferation and tumorigenicity both *in vitro* and *in vivo*

To investigate the effects of AJAP1 on HCC cell proliferation and tumorigenicity, the less invasive SMMC7221 and Huh7 and highly invasive HCCLM3 and SK-Hep-1 cell lines were infected with a lentivirus (LV) expressing short hairpin (sh)RNA targeting AJAP1 (shAJAP1) or encoding AJAP1, respectively. Silencing AJAP1 expression stimulated SMMC7221 and Huh7 cell growth, while AJAP1 overexpression had the opposite effect in HCCLM3 and SK-Hep-1, as determined by growth curve analysis (Figure 2a) and the colony formation assay (Figure 2b). To examine the *in vivo* role of AJAP1, we subcutaneously injected HCC cells into the flanks of nude mice to establish a xenograft tumor model and measured tumor growth. Tumor volume and weight were increased in the SMMC7221-shAJAP1 group as compared to control mice, and were decreased in mice inoculated with HCCLM3-AJAP1 cells (Figure 2c). An immunohistochemical analysis showed that Ki-67 expression was upregulated in the SMMC7221-shAJAP1 group and downregulated in the HCCLM3-AJAP1 group relative to their respective controls (Figure 2d). These results provided the evidence that AJAP1 inhibits HCC cell proliferation and tumorigenicity both *in vitro* and *in vivo*.

### AJAP1 inhibits HCC cell migration, invasion, and lung metastasis

In the wound healing assay, *AJAP1* knockdown enhanced HCC cell migration relative to control cells, whereas AJAP1 overexpression had the opposite effect (Figure 3a). The effects of AJAP1 on HCC cell motility and invasiveness were further evaluated with the transwell migration and Matrigel invasion assays (Figure 3b). SMMC7221 and Huh7 cell migration and invasion were increased upon *AJAP1* knockdown, whereas the opposite was observed in HCCLM3 and SK-Hep-1 cells overexpressing AJAP1.

We then evaluated the role of AJAP1 in tumor metastasis *in vivo* by injecting stably transfected cell lines (SMMC7221-shAJAP1 and HCCLM3-AJAP1) into nude mice via the tail vein and monitoring the development of metastatic nodules in the lungs. Compared to mice, harboring tumors expressing control shRNA (SMMC7221-shCon), mice injected with SMMC7221-shAJAP1 had more and larger lung metastatic nodules. Additionally, tumor mass and number of nodules were lower in the HCCLM3-AJAP1 as compared to the HCCLM3-Con group (Figures 3c and d). The presence of nodules was confirmed by hematoxylin and eosin staining (H&E) of dissected lung tissue (Figure 3e). These results provide further evidence that AJAP1 is involved in the suppression of HCC invasion and metastasis.

### AJAP1 blocks epithelial–to–mesenchymal transition (EMT) in HCC cells

EMT is an important feature of malignant tumors that decreases cell-cell contact and increases migration.^15^ To investigate how AJAP1 controls HCC migration and invasion, we examined the expression of epithelial and mesenchymal markers. A western blot analysis showed that the epithelial markers E-cadherin and zonula occludens-1 were downregulated, whereas the mesenchymal markers N-cadherin and vimentin were upregulated in SMMC7221-shAJAP1 as compared to SMMC7221-shCon cells (Figure 4a). Conversely, AJAP1 overexpression increased epithelial marker expression while repressing that of mesenchymal markers in HCCLM3-AJAP1 cells. These results were confirmed by real-time PCR (Figure 4b) and immunofluorescence (Figure 4c) analyses.

### AJAP1 inhibits EMT by suppressing ZEB1 expression

To clarify the mechanism involved in AJAP1-mediated suppression of EMT in HCC cells, we evaluated the expression of EMT-related transcription factors by real-time PCR. AJAP1 overexpression decreased the level of *ZEB1* but had no effect on the mRNA levels of *Snail*, *Slug*, and *Twist*. On the contrary, *AJAP1* knockdown increased ZEB1 expression without affecting the transcript levels of other EMT-related transcriptional factors (Figure 5a). AJAP1 also decreased ZEB1 and vimentin expression and stimulated that of E-cadherin in HCCLM3 cells, whereas ZEB1 overexpression reversed these effects. Conversely, *AJAP1* silencing resulted in upregulation of ZEB1 and vimentin expression and downregulation of E-cadherin in SMMC7221 cells, whereas *ZEB1* knockdown rescued the decrease in E-cadherin and increase in vimentin expression induced by *AJAP1* silencing (Figures 5b and c), which was confirmed by immunofluorescence analysis (Figure 5d). These results suggest that ZEB1 plays an important role in AJAP1-mediated suppression of EMT in HCC cells.

### ZEB1 is critical for AJAP1-mediated inhibition of HCC cell invasion and metastasis

To further evaluate the role of ZEB1 in AJAP1-mediated inhibition of HCC cell invasion and metastasis, *ZEB1* was knocked down and overexpressed in SMMC7721-shAJAP1 and HCCLM3-AJAP1 cells, respectively. ZEB1 suppression abrogated the increase in SMMC7721 cell migration and invasion resulting from *AJAP1* knockdown, whereas ZEB1 overexpression reversed AJAP1-induced inhibition of migration and invasion in HCCLM3 cells (Figure 6a). To confirm these observations *in vivo*, we monitored tumor metastasis by bioluminescence imaging after injecting luciferase-expressing cells into nude mice via the tail vein. After mice were killed, their lungs were dissected and analyzed by H&E staining. The number of metastatic nodules in the lungs was increased by *AJAP1* silencing, which was reversed by *ZEB1* knockdown. The opposite effects were observed by AJAP1 and ZEB1 overexpression (Figure 6b). These results indicate that ZEB1 is a downstream effector of AJAP1-mediated inhibition of HCC cell invasion and metastasis.

### AJAP1 interacts with and blocks nuclear translocation of *β*-catenin

Since AJAP1 is not a transcription factor, we investigated the molecular basis of AJAP1-mediated ZEB1 inhibition. Wnt/*β*-catenin signaling regulates EMT; given that ZEB1 is a known downstream target of this pathway, we speculated that AJAP1 interacts with *β*-catenin to negatively regulate ZEB1 expression. To test this hypothesis, we co-transfected SMMC7721 and HCCLM3 cell lines with AJAP1 and *β*-catenin constructs, and found that the two proteins interacted (Figure 7a), which was confirmed by an endogenous co-immunoprecipitation (co-IP) assay (Figure 7b) and immunofluorescence analysis (Supplementary Figure 1a). Interestingly, ectopic expression of AJAP1 in HCCLM3 cells increased *β*-catenin accumulation in the cytoplasm while concomitantly reducing its nuclear translocation. Conversely, AJAP1 knockdown in SMMC7721 cells enhanced nuclear translocation of *β*-catenin (Figure 7c and Supplementary Figure 1b).

We used a luciferase reporter assay to determine whether interaction with AJAP1 affects the transcriptional activity of *β*-catenin. Overexpressing AJAP1 attenuated the reporter activity, while *AJAP1* knockdown had the opposite effect (Figure 7d). In the absence of Wnt signaling, *β*-catenin is continually degraded in the cytoplasm; in order to determine how *β*-catenin was protected from degradation and stabilized upon *AJAP1* silencing, we examined the ubiquitination status of *β*-catenin in *AJAP1*-deficient SMMC7721 cells and found that ubiquitination of *β*-catenin was reduced upon *AJAP1* knockdown (Figure 7e), indicating that Wnt signaling could be activated.

We evaluated whether AJAP1-mediated inhibition of ZEB1 is dependent on Wnt signaling by knocking down *β*-catenin in SMMC7721 cells in which AJAP1 was silenced. The upregulation of ZEB1 and vimentin and downregulation of E-cadherin induced by loss of AJAP1 was abrogated and rescued, respectively, by *β*-catenin knockdown (Supplementary Figure 1c). It is possible that AJAP1 forms a complex with *β*-catenin, thereby preventing its nuclear translocation and inhibiting its transcriptional activity (Figure 7f).

### HCC patient prognosis is more accurately predicted by a combination of AJAP1 and ZEB1

Given the reciprocal relationship between AJAP1 and ZEB1, we analyzed their expression in tissue samples from 81 HCC patients by immunohistochemistry, and found a strong negative correlation (*r*=−0.4815, *P*<0.001) (Figures 8a and b). It was previously shown that a combination of molecular markers can improve the prediction of patient prognosis; ^16, 17, 18^ we investigated whether this was the case for AJAP1 and ZEB1 in HCC patients. Indeed, patients with tumors exhibiting low levels of AJAP1 and high levels of ZEB1 had lower survival (Figures 8c and d). Thus, combining AJAP1 and ZEB1 expression improves the prediction of patient outcome.

## Discussion

Hypermethylation of the *AJAP1* promoter has been shown to be a key regulatory mechanism accounting for its altered expression in HCC.^6^ One study found that low *AJAP1* mRNA levels in HCC tissues were associated with poor outcome after curative hepatectomy, particularly for disease-free survival (DFS).^14^ In the present study, we showed that AJAP1 was highly expressed normal liver tissue, and was downregulated with HCC progression. *In vitro* experiments also indicated that AJAP1 expression was negatively correlated with metastasis.

AJAP1 plays an important role in inhibiting tumor cell migration. In the present study, we found that AJAP1 overexpression suppressed tumor formation and lung metastasis of HCC, while *AJAP1* knockdown had the opposite effects. The *in vitro* experiments confirmed that ectopic expression of AJAP1 reduced HCC cell proliferation, tumorigenicity, and metastasis. Accordingly, *AJAP1* knockdown resulted in the upregulation of EMT markers. Among these, expression of the transcription factor ZEB1 was found to be repressed by AJAP1 in HCC, indicating that it mediates AJAP1 suppression of EMT. An analysis of the AJAP1 promoter sequence showed that AJAP1 has putative ZEB1 binding sites. Additional experiments are needed to determine whether ZEB1 regulates AJAP1 transcription, which would suggest a feedback loop between these two factors.

To clarify the regulatory interaction between AJAP1 and ZEB1, we examined the Wnt/*β*-catenin pathway, which is known to regulate ZEB1. AJAP1 forms a complex with E-cadherin and *β*-catenin at cell junctions.^12, 19, 20^ However, it is unclear whether this interaction affects the transcriptional activity of *β*-catenin or has functional implications for HCC. Results of the co-IP assay suggested that AJAP1 interacts with *β*-catenin; moreover, AJAP1 was found to block the nuclear translocation of *β*-catenin and thus, its transcriptional activity. This may be the reason for reduced ZEB1 expression, which could in turn have increased E-cadherin levels and suppressed EMT. These data demonstrate that the AJAP1/*β*-catenin complex represses ZEB1 and prevents HCC metastasis. The immunohistochemical analysis of HCC specimens confirmed an association between AJAP1 and ZEB1. In addition, we found that the combination of AJAP1 and ZEB1 expression had better prognostic value for DFS and overall survival of HCC patients.

In conclusion, we identified AJAP1 as a key regulator of HCC progression and provided evidence for a novel AJAP1/*β*-catenin/ZEB1 signaling axis in the regulation of HCC carcinogenesis and metastasis. These findings indicate that AJAP1 can serve as a prognostic biomarker and therapeutic target for HCC treatment.

## Materials and Methods

### Cell lines and reagents

The L02 immortalized liver cell line was purchased from the Institute of Biochemistry and Cell Biology, Chinese Academy of Science, China. SMMC7721, Huh7, HCCLM3, and Sk-Hep-1 human HCC cells were purchased from the American Type Culture Collection (Manassas, VA, USA), and MHCC97L and MHCC97H metastatic human HCC cell lines were obtained from the Liver Cancer Institute and Zhongshan Hospital of Fudan University, Shanghai, China. Cells were cultured at 37 °C and 5% CO_2_ in Dulbecco's modified Eagle's medium supplemented with 10% fetal bovine serum and 1% antibiotics (100 U/ml penicillin and 100 *μ*g/ml streptomycin). An LV vector encoding the human AJAP1 gene (LV-AJAP1) was constructed using FUW-teto (Addgene, Cambridge, MA, USA); the empty vector (LV-control) was used as a negative control. LV-shAJAP1, LV-ZEB1, and LV-shZEB1 were constructed in the same manner. All LV vectors, including one encoding the human firefly luciferase gene, were generated by GeneChem Technologies (Shanghai, China). HCC cells were transfected with the LV vectors and selected starting 48 h later for 2 weeks with 2 *μ*g/ml puromycin (Sigma-Aldrich, St. Louis, MO, USA). Pooled populations of transfected cells collected 2 weeks after drug selection without subcloning were used for *in vitro* and *in vivo* experiments. MG132 was purchased from Selleck Chemicals (Houston, TX, USA). Primary antibodies and dilutions used in this study are listed in Supplementary Table S1. Primers used for real-time PCR are listed in Supplementary Table S2.

### HCC tissue collection

A total of 81 HCC patients were enrolled in this study. Archival HCC tissue samples were collected from patients who underwent HCC resection from January 2008 to May 2013 at the First Affiliated Hospital of Harbin Medical University. HCC diagnosis was based on World Health Organization criteria. Clinical typing of tumors was according to the International Union against Cancer tumor-node-metastasis classification system. Liver function was assessed according to the Child-Pugh scoring system. Tumor differentiation was defined according to the Edmondson grading system. Ethical approval for the use of human specimens was obtained from the Research Ethics Committee of the First Affiliated Hospital of Harbin Medical University. Patients provided written, informed consent. Detailed characteristics of the 81 paired specimens are summarized in Supplementary Table S3.

### Tissue microarray and immunohistochemistry

Normal and cancerous human liver tissue microarrays (BC03119a) were obtained from U.S. Biomax (Rockville, MD, USA). AJAP1 and Ki-67 expression in tumor tissues was detected by immunohistochemistry as previously described.^18^

### Real-time PCR

Total RNA was extracted from cultured cells using the RNAeasy Mini kit (Qiagen, Valencia, CA, USA) according to the manufacturer's instructions. Reverse transcription was performed using the High Capacity Reverse Transcription kit (Applied Biosystems, Foster City, CA, USA) after RNA quantification. Real-time PCR was performed using the Power SYBR Green PCR Master Mix (Life Technologies, Carlsbad, CA, USA) or TaqMan Fast Universal PCR Master Mix on an ABI Prism 7900HT instrument (Applied Biosystems). Expression levels of target genes were normalized to that of glyceraldehyde 3-phosphate dehydrogenase and determined according to the 2^−ΔΔCt^ method.

### Cell growth and colony formation assay

HCC cells (5 × 10^4^ per well) were seeded in 6-well plates. The number of viable cells was counted at different time points. For the colony formation assay, cells were seeded in 6-well plates at a density of 500–800 cells per well and cultured for 14 days. Colonies were stained with 0.5% Crystal Violet for 10 min and counted.

### Wound healing assay

Cells were cultured in a 6-well plate and grown to confluence. Cells were washed three times with the medium and the bottom of well was scratched with a 200- *μ*l pipette tip. Images were captured at 0 and 24 h on an Eclipse TS100 microscope (Nikon, Tokyo, Japan).

### Cell migration and invasion assays

To evaluate cell migration, 2–4 × 10^4^ cells were seeded in the upper chamber of the transwell insert in serum-free medium and migration at 37 °C towards normal medium was evaluated after 24 h. The cell invasion assay was performed using Matrigel-coated membranes (BD Biosciences, Franklin Lakes, NJ, USA) in 24-well dishes. The assay was carried out for 24–48 h at 37 °C. Cells that migrated through the membrane filter were fixed in methanol, stained with 0.5% Crystal Violet in methanol, and counted under the light microscope. Each experiment was performed in triplicate. Cells that migrated to the lower side of the filters (that is, invaded cells) were counted at 200 × magnification in five different microscopic fields per filter.

### Western blotting

Whole cell or tissue extracts were prepared in radioimmunoprecipitation assay buffer containing protease and phosphatase inhibitors. After determining the concentration, 30 *μ*g of protein were denatured and resolved by sodium dodecyl sulfate polyacrylamide gel electrophoresis and then transferred to a polyvinylidene fluoride membrane (Invitrogen, Carlsbad, CA, USA) that was blocked with 5% skim milk and incubated with primary antibodies overnight at 4 °C. The membrane was then incubated with alkaline phosphatase-conjugated secondary antibodies, and protein bands were visualized by enhanced chemiluminescence (Pierce, Rockford, IL, USA).

### Immunofluorescence (IF)

The day before the experiment, HCC cells were seeded on glass slides and fixed in 4% paraformaldehyde, followed by permeabilization with 0.5% Triton X-100 for 15 min. After washing with phosphate-buffered saline (PBS), cells were blocked with 10% normal goat serum for 30 min and then incubated overnight at 4 °C with primary antibodies. The cells were washed with PBS and incubated with Alexa Fluor 488- or 555-conjugated secondary antibodies for 1 h at room temperature; nuclei were stained with 4',6-diamidino-2-phenylindole (Vector Laboratories, Burlingame, CA, USA), and images were captured with a DMRA fluorescence microscope (Leica, Wetzlar, Germany).

### Co-IP assay

Cells were treated with MG132 (20 *μ*M) for 8 h, harvested, and lysed in 400 *μ*l co-IP buffer containing a protease inhibitors cocktail (Sigma-Aldrich). The lysate was centrifuged and the supernatant was precleared by incubation with 20 *μ*l immobilized protein A/G beads (Santa Cruz Biotechnology, Santa Cruz, CA, USA) for 1 h at 4 °C, followed by overnight incubation at 4 °C with 20 *μ*l anti-AJAP1 antibody or control IgG. Protein complexes were precipitated by incubation with 30 *μ*l immobilized protein A/G beads for 2 h at 4 °C. Samples were washed four times with lysis buffer; the beads were boiled in loading buffer, and proteins were detected by western blotting.

### Luciferase assays

Cells (5 × 10^4^) were seeded in 24-well plates and cultured for 24 h. Cells were transfected with 200 ng TOP/FOP reporter luciferase plasmid (GeneChem Technologies, Shanghai, China), and 10 ng of pRL Renilla luciferase (as an internal control) using Lipofectamine 2000 (Invitrogen) according to the manufacturer's instructions. Cells were subjected to luciferase reporter assay 24 h after transfection, using the Dual-Luciferase Reporter Assay System (Promega, Madison, WI, USA).

### Animal studies

Male BALB/c athymic nude mice (4–6 weeks old) were purchased from the experimental animal center of Shanghai Institute for Biological Sciences. Mice were housed under standard conditions and maintained according to the institutional guidelines for animal care. To establish a subcutaneous xenograft model, 2 × 10^6^ cells in 100 *μ*l PBS were subcutaneously injected into the flank of mice. Tumors were removed after 4 weeks, and their size and weight were determined. The experimental metastasis model was established by injecting 4 × 10^6^ cells into the tail vein of nude mice (10 per group). After 8 weeks, metastatic tumors were imaged with the NightOWL LB983 system (Berthold Technologies, Wildbad, Germany) following D-luciferin (Promega) injection. Animal procedures were authorized by the Institutional Animal Care and Use Committee of Harbin Medical University.

### Statistical analysis

Results are presented as mean±S.D. Multiple groups were compared by one-way analysis of variance followed by Dunnett's *t*-test. A *P*-value<0.05 was considered statistically significant.

## Figures and Tables

**Figure 1:** AJAP1 is downregulated in human HCC and negatively correlates with metastasis of HCC. (**a**) Representative immunohistochemical detection of AJAP1 in tissue microarrays of normal liver tissue and different grades of HCC. Scale bar=100 *μ*m. (**b**) Percentage of patients with high and low AJAP1 expression according to the following clinical parameters: tumor size (cm), tumor stage (I–II and III–IV), lymph node status (N0 or N1), and metastasis status (M0 or M1). (**c**) Western blot analysis of HCC and matched non-tumorous tissues from a different cohort. (**d**) Western blot analysis of AJAP1 expression in L02 and various HCC cell lines, and relative *AJAP1* mRNA levels in L02 and HCC cell lines as detected by real-time PCR. The data are expressed as mean±S.D. of three independent experiments. *P<0.05; **P<0.01; ***P<0.001. T: tumor; N: normal tissue

**Figure 2:** AJAP1 suppresses HCC cell growth *in vitro* and *in vivo*. (**a**) Growth curves were generated based on counts of indicated HCC cells (shCon, shAJAP1, Con, and AJAP1). (**b**) Results of the colony formation assay with HCC cells are shown in the upper panels. Number of foci was counted as shown in the lower panels. (**c**) *AJAP1* knockdown increases SMMC7221 cell xenograft growth in nude mice, while AJAP1 overexpression decreases HCCLM3 cell xenograft growth in nude mice. Tumor volume and weight are shown. (**d**) AJAP1 and Ki-67 expression as detected by immunohistochemistry. Scale bar=25 *μ*m. The data are expressed as mean±S.D. of three independent experiments. *P<0.05; **P<0.01; ***P<0.001

**Figure 3:** AJAP1 inhibits HCC cell migration and lung metastasis. (**a**) Representative image from the wound healing assay (left panel). *AJAP1* knockdown with LV-shAJAP1 enhanced SMMC7721 and Huh7 cell migration *in vitro*, whereas AJAP1 overexpression with LV-AJAP1 suppressed HCCLM3 and SK-Hep-1 cell migration. Representative images were obtained at 0 and 24 h after scratching, and wound closure was quantified by measuring the area without migrated cells using ImageJ software (National Institutes of Health, Bethesda, MD, USA) (right panel). Scale bar*=*200 *μ*m. (**b**) Representative images of migration and invasion assays for HCC cell lines. (**c**) *In vivo* metastasis assay using stably transfected cell lines injected into nude mice via the tail vein and representative images of the lungs of mice. (**d**) Number of lung metastatic nodules in each group. (**e**) Representative images of lung tissue samples from different experimental groups after H&E staining of lung metastatic nodules (*n=*10/group). Scale bars*=*500 *μ*m. The data are expressed as mean±S.D. of three independent experiments. *P<0.05; **P<0.01; ***P<0.001

**Figure 4:** AJAP1 blocks EMT in HCC cells. (**a**) AJAP1, E-cadherin, zonula occludens (ZO)-1, N-cadherin, and vimentin expression was evaluated by western blotting in SMMC7721 and HCCLM3 cells (shCon, shAJAP1, Con, and AJAP1). (**b**) Expression of EMT markers after ectopic expression of AJAP1, as determined by real-time PCR. (**c**) Immunofluorescence analysis of E-cadherin and vimentin expression in SMMC7721 and HCCLM3 cells. The data are expressed as mean±S.D. of three independent experiments. *P<0.05; **P<0.01; ***P<0.001

**Figure 5:** AJAP1 blocks EMT via regulation of ZEB1 expression. (**a**) Effect of AJAP1 overexpression (upper panel) or knockdown (lower panel) on the expression of ZEB1, Snail, Slug, and Twist, as evaluated by real-time PCR. (**b** and **c**) Western blot and real-time PCR analyses of AJAP1, ZEB1, E-cadherin, and vimentin expression. ZEB1 overexpression using LV-ZEB1 abrogated the increase in E-cadherin expression induced by AJAP1. Conversely, *ZEB1* knockdown using LV-shZEB1 reversed the downregulation of E-cadherin in SMMC7721-shAJAP1 cells. (**d**) Immunofluorescence analysis of E-cadherin and vimentin expression in HCC. The data are expressed as mean ± S.D. of three independent experiments. *P<0.05; **P<0.01

**Figure 6:** ZEB1 is critical for AJAP1-mediated inhibition of HCC invasion and metastasis. (**a**) Cell migration and invasion were assessed with the transwell assay. *ZEB1* knockdown decreased *AJAP1* knockdown-induced cell migration and invasion in SMMC7721 cells, whereas ZEB1 overexpression had the opposite effect in HCCLM3 cells. The right panel shows the counts of migrated and invaded cells. (**b**) Bioluminescence imaging of lung metastasis. Cell lines stably expressing luciferase (SMMC7721-shAJAP1 and SMMC7721-shAJAP1 plus LV-shZEB1; HCCLM3-AJAP1 and HCCLM3-AJAP1 plus ZEB1; and their respective controls) were injected into mice via the tail vein, and luciferase activity was monitored. (**c**) Incidence of lung metastasis in each group was counted. (**d**) Histological analysis of lung tissue samples from different groups by H&E staining. The data are expressed as mean±S.D. of three independent experiments. *P<0.05; **P<0.01

**Figure 7:** AJAP1 interacts with and inhibits nuclear translocation of *β*-catenin. (**a**) Results of the co-IP assay showing that AJAP1 forms a complex with *β*-catenin in both SMMC7721 and HCCLM3 cells. (**b**) Reciprocal co-IP of endogenous proteins showing a strong interaction between AJAP1 and *β*-catenin. (**c**) AJAP1 overexpression inhibits nuclear translocation of *β*-catenin, while *AJAP1* knockdown has the opposite effect. (**d**) AJAP1 overexpression suppressed whereas AJAP1 silencing enhanced TOPflash reporter activity, respectively. (**d**) Ubiquitination of *β*-catenin is reduced upon *AJAP1* knockdown. (**e**) In normal tissue, AJAP1 interacts with *β*-catenin and inhibits its nuclear translocation, thereby suppressing *β*-catenin-induced ZEB1 activation and inhibiting HCC carcinogenesis and metastasis. In HCC, AJAP1 is silenced; *β*-catenin translocates to the nucleus to activate ZEB1 transcription, leading to HCC progression. The data are expressed as mean ± S.D. of three independent experiments. *P<0.05; **P<0.01

**Figure 8:** Combination of AJAP1 and ZEB1 better predicts HCC patient prognosis than either factor alone. (**a**) Correlation between AJAP1 and ZEB1 levels analyzed in 81 patients by immunohistochemistry. (**b**) Representative images of AJAP1 and ZEB1 expression. (**c** and **d**) Kaplan–Meier analysis of overall survival and DFS in patients with variable expression of AJAP1 and ZEB1.
